# “Before Dawn,” Listening to the Voices of Social Media: A Study on the Public's Response to the COVID-19 Vaccine

**DOI:** 10.1155/2022/7308084

**Published:** 2022-09-16

**Authors:** Jiangyi He, Maojun Zhou

**Affiliations:** School of Journalism and Communication, Wuhan University, Wuhan 430072, China

## Abstract

The COVID-19 pandemic is a worldwide catastrophe. In the absence of an effective drug, one effective measure to pull the pandemic to the end is herd immunity by taking vaccines, while the hesitation and anti-attitude from social media affect the vaccination. This makes it crucial to evaluate the text data about the COVID-19 vaccine from tweets. The period for data used in this study is 1 Aug to 31 Oct, 2020, since it is just before promoting the use when public reactions to the COVID-19 vaccine can influence their subsequent vaccination behavior. In this study, we used the latent Dirichlet allocation (LDA) topic model and sentiment analysis to explore public reactions to the COVID-19 vaccine. The results indicate that the public discussion could be divided into 11 topics, which could be further summarized into four different themes: (1) concerns about COVID-19; (2) concerns about vaccine development, production, and distribution; (3) how to control the COVID-19 before obtaining the vaccine; and (4) concerns about information of vaccine safety and efficacy. It can be concluded that to a large extent, public reactions to vaccines are dominated by positive sentiment. Specifically, the politicization of the vaccine approval process, suspension of vaccine trials, and measures to control COVID-19 tend to trigger negative public sentiment; whereas information related to successful vaccine development and availability enhances positive public sentiment. These findings help us understand public reactions to the COVID-19 vaccine, uncover potential factors that may influence vaccination behavior, and help policymakers understand public opinion about the COVID-19 vaccine and develop rational and effective policies.

## 1. Introduction

The disease caused by the SARS-CoV-2 virus was named coronavirus disease 2019 (COVID-19) by the World Health Organization (WHO) in February 2020, which has spread rapidly and become an international pandemic after its discovery. Until December 21, 2021, reported data from WHO show that there are 270 million confirmed cases and more than 5.35 million deaths worldwide [1]. To end the epidemic, several interventions are adopted, such as wearing masks, lockdowns, quarantines, social distancing, and frequent hand washing. However, these methods have limited success, with large numbers of people committing or dying from COVID-19. The risk of reinfection and strain mutation makes it increasingly difficult to end a pandemic in a short period of time. The socioeconomic impact of COVID-19 is now far greater than that of severe acute respiratory syndrome (SARS) and the Middle East respiratory syndrome (MERS) [2], and the rate of infection and mortality caused by COVID-19 has far exceeded that of other influenzas [3]. COVID-19 has become a public health emergency on a global scale.

It has become a global expectation to end the pandemic as soon as possible to facilitate the return of economic order and social life to normal. In the absence of effective drugs, the development of a safe and effective vaccine and immunization through vaccination are considered the two most effective measures to prevent the further spread of the epidemic. Therefore, scientists around the world have launched a race to develop a vaccine. Although Russia first announced the approval of the world's first COVID-19 vaccine (Sputnik V) on August 11, 2020, the vaccine was not in Phase III clinical trials and was only available to a limited population. Till November, a growing number of pharmaceutical companies announced that they had developed a vaccine with high efficacy and received emergency access subsequently. However, a safe and effective COVID-19 vaccine still remains unavailable in most countries and regions of the world on a global scale, when this period is considered to be “pre-dawn.” While the successful development of the vaccine holds promise for containing the development of the pandemic, potentially influential factors for vaccination still exist, such as vaccine hesitation and anti-vaccine. For example, it is shown that more than 70% of working-age people will refuse the COVID-19 vaccine or remain hesitant in France [4]. Survey data from the U.S. indicates that acceptance of vaccines was above 72% in April 2020, but dropped to 48% in October [5]. Murphy's results show that 26% of Irish respondents and 25% of UK respondents were hesitant to take the vaccine [6]. This makes it important to study the public's response to the COVID-19 vaccine.

Text analysis of tweets (including topic modeling and sentiment analysis) has become one of the important directions of information epidemiology research. For the public, social media has become an important online venue for public opinion expression. Tweets from the Internet are not only the digital footprints of Internet users but also the reproduction of their “voices in the cloud,” which reflect the public's reactions to specific events. Moreover, public reactions may have a contagious effect on the attitudes and behaviors of other social media users. As a globally influential social media platform, Twitter had 206 million profitable daily active users worldwide by the second quarter of 2021 [7]. During the pandemic, the personal activity of the public on Twitter increased significantly. Therefore Twitter can be considered a valuable information platform that can be used to dynamically track and assess public discussion and attitudes towards the COVID-19 vaccine.

It is particularly important to study the public response to COVID-19 vaccine before the “twilight,” since the public's reaction to the vaccine during this period is closely related to subsequent vaccination behavior. In this study, we analyzed tweets about the COVID-19 vaccine using mainly topic modeling and sentiment analysis. The objectives of this study include: first, to explore topics of public interest and changes in public sentiment toward the COVID-19 vaccine to help us assess public response to the vaccine and uncover potential factors that may influence vaccination; second, to help policymakers develop more effective communication, education, and policy implementation strategies [8] to increase public acceptance of the COVID-19 vaccine by using Digital Health [9]; third, to provide experience learned for pandemics caused by other unknown viruses; and fourth, to help decision makers understand the public opinion trends regarding COVID-19 vaccine and avoid outbreaks of vicious mass events.

## 2. Materials and Methods

### 2.1. Data Collection

In this study, we selected vaccine-related tweets on Twitter as a corpus and performed topic modeling and sentiment analysis. There are two main reasons for Twitter to be selected: (1) as the “message on the Internet,” it is a widely and freely used social platform in the world; (2) it is more open than other social platforms such as Facebook where everyone can access most of its content [10]. The data for this article comes from tweet data about the novel 2019 coronavirus provided by The George Washington University library: the data contains multiple hashtags (e.g., #Coronavirus, #COVID19, #CoronaOutbreak) by Kerchner and Wrubel, and contains tweet data from various countries worldwide [11]. First, using vaccine and vaccination as keywords, the data are filtered and restricted to the period August 1 to October 31, 2020, based on the search tool provided by George Washington University. This time period is crucial for observing public reactions to the vaccine on social media due to three aspects: first, the global epidemic has entered a high outbreak stage; second, scientists in various countries have also launched a race to develop vaccines; and third, this time period is before the successful vaccine development. The systematic sampling method is conducted on the obtained data, together with repeated sampling. Since English is the most widely spoken language worldwide, only English texts were selected for analysis.

In addition, we compared the text data of all tweets and obtained a total of 37,688 tweets after removing duplicate data. It should be noticed that we cannot obtain any information about tweets of the logouts and those deleted by the user due to the restrictions of Twitter's company policy. Finally, we store the obtained metadata (e.g., tweet text, creation time) in a database. The final dataset size is 37,688 ∗ 2 = 75,376.

### 2.2. Data Preprocessing

Before topic modeling and sentiment analysis, the collected text data is pre-processed. First, the extraction, cleaning of the data and character removal are realized by pandas and re libraries in Python. In this step, the removals include Url, Emojis, retweet marks (e.g. RT), mention marks (e.g. @), hashtags (e.g. #), e-mail addresses, line breaks, punctuation marks, and other meaningless characters (e.g. amp) that may be contained in the tweets. Another preprocessing procedure is word splitting. Before that, all tweets are converted to lowercase using the lower() function. Based on spaCy, word tokenization (the nouns, adjectives, verbs, and adverbs are retained) and lemmatization (e.g., was to be) are operated. Stop words contained in the tweets are also removed.

### 2.3. Temporal Analysis

To understand the temporal-level trends of tweets, we focused on the temporal analysis of all tweets from August 1 to October 31, 2020, which includes: (1) temporal trends in the number of tweets; (2) temporal trends in the number of topics; (3) temporal trends in the sentiment of tweets; and (4) temporal trends in the sentiment of tweets under different topics.

### 2.4. Topic Analysis

Traditional text analysis techniques are based on coding, but there are some obvious drawbacks. For example, the coding process relies on the researcher's prior knowledge and it is time-consuming and costly. This drawback was not yet prominent when the sample size is small; as the sample size increased, the drawbacks of manual coding become increasingly apparent. With the large sample data, researchers began to consider using topic models in unsupervised machine learning to analyze text data. In topic modeling, words and documents are connected by topics, which means that each topic corresponds to multiple word distributions and each document corresponds to pairs of topics. As a mainstream approach in topic modeling, Latent Dirichlet Allocation (LDA) was first proposed by Blei et al. [12]. And the LDA model was improved by Griffiths and Steyvers in 2004 [13]. LDA has been widely used in social science research. For example, Xue et al. used LDA to analyze Twitter data to understand public discourse on social media during pandemics [14]; Liu et al. used online pharmacy reviews as data to explore potential factors influencing consumer satisfaction [15]; Scarborough and Helmuth et al. used LDA models to map the cultural reputation of cities [16]. In this study, LDA is conducted by Gensim to model the themes of tweet data after a bigram model and document-terminology matrix construction.

### 2.5. Sentiment Analysis

Text data from the Internet (e.g., information on social media, user reviews of goods and services) is considered as an online expression of public sentiment. The purpose of sentiment analysis is to score or classify textual data by automatic analysis for public attitudes toward specific events, products, people, and other objects. In social science such as business, politics, and public action [17], sentiment analysis has become a more popular text mining method. In business, researchers typically analyze the relationship between sentiment from reviews on the Internet and product sales [18, 19]. In the political domain, Tumasjan et al. found that the sentiment of tweets is closely related to the positions of politicians [20]. In the field of public action, sentiment can also be used to monitor the occurrence of collective social action [10]. In the field of communication, El Barachi et al. used sentiment analysis to gain insight into the direction of public opinion on social media [21], Gu et al. used Sina Weibo texts as data to explore changes in user sentiment on social media during emergencies [22] while Wang et al. evaluated sentiment on social media rumors during epidemics [23].

It seems that Python and R have become important tools for researchers to perform sentiment analysis [24], and several modules related to sentiment analysis have been developed, such as syuzhet, RSentiment, SentimentR, SentimentAnalysis, and meanr in R and Textblob and VADER in Python. Compared to other packages in R, SentimentR has good runtime performance and the lowest misclassification rate in terms of accuracy [25]. Considering that VADER has higher accuracy than Textblob in analyzing social media texts and similar results to SentimentR in sentiment recognition [26], thus this study uses SentimentR package to score vaccine tweets [27].

## 3. Results

### 3.1. Tweet Analysis

*Temporal Trends of Tweets*.  Figure 1 reflects the trend of the number of tweets related to the COVID-19 vaccine.  Table 1 shows the ten highest number of tweets posted with their corresponding date. Overall, the number of tweets fluctuated widely. There are two days with their daily posts exceeding 1,000, while the lowest number of tweets is 160 on October 10. In general, the number of tweets was at its peak on weekdays with more focus on vaccine, and at its trough on weekends with less concern about the vaccine (Figure 2). Specifically, Tuesday had the highest number of tweets at 7,062, followed by Thursday (*N* = 6,699), Wednesday (*N* = 6,671), Friday (*N* = 5,388), and Monday (*N* = 5,026); Saturday (*N* = 3,698) and Sunday (*N* = 3,144) had the lowest number of tweets. This phenomenon is also known as the “Fresh start effect,” when people are more likely to pursue various aspirational behaviors at the beginning of the week [28], leading to a higher level of public interest in vaccines.

*Word Frequency*. Word frequency, to a certain extent, reflects the degree of public attention to a specific topic on social media. Ranking the frequency of keywords in descending order, Figure 3(a) shows that the 10 most frequent keywords include trials (*N* = 4,724), say (*N* = 3,918), get (*N* = 2,812), COVID (*N* = 2,723), people (*N* = 2,566), first (*N* = 1,937), vaccine (*N* = 1,934), take (*N* = 1,918), need (*N* = 1,731), and develop (*N* = 1,715). This study used Python's WordCloud library to plot the word cloud (Figure 4). The larger font of the word indicates the more frequently the term appears in the tweets. The word cloud map shows that topics related to the vaccine trial (including the progress of the trial and public reaction to the trial) and the development of the outbreak were the most popular topics.

*Bigrams*. The Bigrams is an ordered arrangement of two words in a document. Based on the words in the list, this study constructed bigrams of words.  Figure 3(b) shows the ten most frequently occurring Bigrams including: “herd immunity, million doses, serum institute, phase iii, sars cov, unexplained illness, side effects, Oxford university, emergency use, bill gates.” The Bigrams indicate that the discussion about the vaccine is mainly related to the public's concern about COVID-19 symptoms, and expectations or concerns about the vaccine. Meanwhile, the “bill gates” in the Bigrams indicates the public's concern about celebrities. This is mainly in two aspects: first, the concern about the Gates Foundation's involvement in vaccine development, due to the efforts of Bill Gates and his foundation in the production, promotion and vaccination of vaccines; second, resistance to the Gates Foundation's involvement in the development of vaccines, due to the news that the vaccines involved and developed by Gates Foundation may alter human DNA.

In order to analyze the content of the tweets in more depth, we use the LDA model to perform topic modeling analysis on the collected tweets and SentimentR to perform sentiment analysis on the tweets in the following section.

### 3.2. Topic Modeling

In order to find the optimal number of topics, we use coherence as a model selection index for model evaluation, since it is a good indicator of the interpretability of the topic model [29, 30]. A larger consistency score means better prediction performance of the model. First, we estimated 20 topic models (starting from *K* = 2 with a step size of 3).  Figure 5(a) shows the consistency scores corresponding to each topic model. The consistency score increases as *K* increases, and then the trend of the consistency score increases slowly with a fluctuated characteristic afterward. The consistency score of the topic model is highest when *K* = 11. Then, we estimated seven more topic models (from *K* = 8 to *K* = 14 with a step size of 1). The line chart of the consistency scores is shown in Figure 5(b) below, where the consistency score is highest when *K* = 11. Therefore, we determined the optimal number of topics to be 11.

We select 15 key terms and representative documents under each topic for concept extraction and explanation of the topic.  Table 2 and Figure 6 reflect the key terms corresponding to different topics and their probabilities in the topic distribution, respectively.  Figure 7 reflects the frequency distribution of tweets under each topic. The highest attention was paid to Topic 3 (*N* = 4,551), accounting for 12.08% of the total number of tweets, followed by Topic 0 (*N* = 4,297), accounting for 11.40% of the total number of tweets, and the lowest attention was paid to Topic 9 (*N* = 2,495), accounting for 6.62% of the total number of tweets.

#### 3.2.1. Related Topics and Themes

Topic 0 deals with the coverage and discussion of the equitable distribution of vaccines globally. This equity does not only refer to the distribution among countries (rich vs. poor), regions (urban vs. rural), races (colored or white) and genders, but also focuses on vulnerable populations (e.g., the homeless). For example, several countries, including China, Canada, and the United Kingdom, have joined the COVAX program promoted by WHO to ensure the equitable distribution of vaccines worldwide. In addition, it is also considered by some people that vaccines are public goods which need to be wary of “vaccine nationalism.” Vaccine nationalism can lead to hoarding of the vaccine and higher prices, and even prolong the duration of pandemics. Related keywords include health, pandemic, global, public, ensure, include, part, effort, access, support, fight, expert, response, lead, and group.

Topic 1 involves a discussion of control measures prior to obtaining a vaccine, including both social measures (e.g., wearing masks, blockades) and immunization measures (e.g., cross-immunization, herd immunization). These discussions involve not only warnings (e.g., “be wary of mental exhaustion before obtaining the vaccine and forgo using social measures.”) but also rumors (e.g., “Just like with smokers, coal miners be immune to COVID-19 ...”). In addition, some members of the public have expressed concern about “herd immunity,” suggesting that herd immunity through disease transmission would lead to more deaths. Related keywords include virus, time, spread, infection, mask, patient, immunity, population, disease, control, show, kill, close, long, and rate.

Topic 2 refers to conversations between professionals and the public about vaccine knowledge. These conversations include coverage and discussion of the latest developments in vaccine research, vaccine outlook, safety and efficacy, misinformation about vaccine coverage, vaccine hesitancy, and how to eliminate vaccine stigma around the COVID-19 vaccine. Related keywords include read, research, development, late, great, live, update, question, talk, join, share, discuss, watch, learn, and challenge.

Topic 3 covers the progress of the vaccine clinical trials. One of the more discussed topics was related to the suspected adverse reactions in UK participants and the forced stoppage of the phase 3 study of the AstraZeneca vaccine. In addition, other vaccines were also discussed. For example, phase 1 and phase 2 clinical trials of an inactivated vaccine developed in China showed positive results according to a study published in the Journal of the American Academy. Related keywords include trial, clinical, phase, candidate, study, volunteer, start, early, AstraZeneca, human, begin, result, show, pause, and participant.

Topic 4 addresses the politicization of the vaccine approval process and the crisis of confidence in vaccines. For example, some members of the public believed that Trump's early false statements (e.g., that the virus would eventually go away, that the disinfectant could cure the virus) were related to the further spread of the outbreak across the United States. This has also led to a crisis of public confidence in President Trump. In addition, because of the approaching election it is concerned that political factors may play a role in the approval process of the vaccine. Some critics claim that the pandemic should not be viewed as a partisan issue and reject the use of unproven vaccines that lack scientific data. Instead, the public has shown a high level of trust in Dr. Anthony Fauci and claims to trust the CDC only if Dr. Fauci claims the vaccine is legal, safe, and effective. Related keywords include make, trump, election, trust, science, rush, official, top, speed, push, big, explain, clear, pay, and political.

Topic 5 deals with governments' plans for vaccine procurement (trading), and distribution. The related topics involve various countries such as the United States, Canada, Australia, and India. As a regional organization, the EU is committed to providing vaccines to its member states. Related keywords include plan, end, government, state, ready, free, announce, dose, potential, sign, promise, provide, deal, supply, and distribution.

Topic 6 involves discussions of the twindemic of influenza and COVID-19 pandemic. For example, these discussions include concerns about coinfection with influenza viruses and COVID-19 viruses; recommendations for people to receive influenza vaccines to reduce the risk of influenza infection and reduce the burden on the health care system; reminders that influenza vaccines are neither effective in preventing COVID-19 nor in increasing the risk of infection; and information about mandating vaccination for children ages 3–18 by U.S. pharmacists. Related keywords include year, flu, find, people, important, protect, good, risk, covid, child, shot, time, prevent, vaccinate, and increase.

Topic 7 involves a discussion of virus testing prior to obtaining a vaccine. Testing for the virus is used to ensure people's safety in order to facilitate the reopening of schools, the recovery of the economy, and the return of life to normal. Related keywords include test, give, people, back, life, hope, thing, care, call, school, lie, cure, vote, positive, and open.

Topic 8 focuses primarily on concerns about the safety and efficacy of vaccines. For example, the public has called for ensuring transparency, science, and rigor in the vaccine review process. Vaccine companies (pharmaceutical companies) have pledged not to seek premature approval from the government without extensive safety and efficacy data, and senior FDA scientists have pledged not to approve vaccines under political pressure. The safety and efficacy of Sputnik V, a vaccine from Russia, have been called into question because scientific data on vaccine testing has not been released. Related keywords include coronavirus, news, safety, race, datum, receive, treatment, Russian, approval, follow, drug, base, good, release, and expect.

Topic 9 addresses concerns about the development of COVID-19 (e.g., total confirmed cases, new cases in a single day, new deaths in a single day). At the same time, the public is questioning herd immunization measures due to the emergence of reinfection cases and the rising number of confirmed cases and deaths. Related keywords include covid, people, case, day, report, month, death, week, die, wait, stop, high, happen, strategy, and bad.

Topic 10 deals with advocating for a collaborative effort to develop a safe and effective vaccine to end a pandemic. The production of vaccines is a globally collaborative process. For example, the development of a vaccine may be done in country A, while the bottles that contain the vaccine may be produced in country B, and the glass used to produce the bottles may come from country C. This requires increased global collaboration to address COVID-19. Related keywords include vaccine, develop, world, work, safe, country, effective, covid, scientist, approve, produce, create, make, deliver, and development.

Finally, we used a qualitative approach to divide the 11 topics into 4 different themes (as shown in Table 2): Theme 1 deals with concerns about COVID-19 (topics 6 and 9); Theme 2 deals with vaccine development, production, and distribution (topics 0, 3, 5, and 10); Theme 3 relates to the control of outbreak before obtaining the vaccine (topics 1 and 7); and Theme 4 covers knowledge or information about vaccine safety and efficacy (topics 2, 4, and 8).

#### 3.2.2. Temporal Trends in Topics

Figure 8 reflects the temporal trend of the number of tweets under each topic. Except for the four peak periods, the change in topic counts is moderate at other times. Peak 1 occurred on August 11, with 295 tweets for topic 10. Peak 2 occurred on September 9, with 349 tweets for topic 3. Peak 3 occurred on October 13, with 229 tweets for topic 3. Peak 4 occurred on October 22, with 309 tweets for topic 5. In general, these spikes are associated with the “Fresh start effect” on the one hand, and public interest in vaccine development, production, and distribution on the other hand. The August 11 opinion spike was related to Russia's approval of the world's first COVID-19 vaccine; the September 9 opinion spike was related to the suspension of clinical trials for the AstraZeneca vaccine; the October 13 opinion spike was related to Johnson & Johnson's suspension of vaccine trials; and the October 22 opinion spike was related to the BJP's vaccine supply pledge.

### 3.3. Sentiment Analysis

In this section, we use the SentimentR package in R to rate the sentiment of each tweet. The maximum value of the sentiment score is 1.725, which means that the tweet expresses the most positive sentiment, and the minimum value of the sentiment score is −2.062, which means that the tweet expresses the most negative sentiment. The mean and median of sentiment scores were 0.073 and 0.056, respectively. Based on the sentiment scores, we classified the tweets into three categories: positive sentiment (score > 0.1), neutral sentiment (−0.1 ≤ score ≤ 0.1), and negative sentiment (score < −0.1). Among them, positive sentiment (*N* = 16,589) accounted for the largest share, about 44.02%, followed by neutral sentiment (*N* = 12,475), about 33.10%, and the smallest share of negative sentiment (*N* = 8,624), about 22.88%.

Figure 9 reflects the trend of the sentiment score over different time periods. The sentiment score of a single day is calculated as the average of the sentiment scores of all tweets on that day. From the figure, the sentiment varies widely across time, but there are four distinct trough periods (sentiment scores less than 0.02). The average sentiment score was 0.0136 on August 2, 0.0157 on August 22, 0.0084 on September 9, and −0.0090 on October 13. In order to further illustrate the reasons for the emergence of low mood periods, we separately calculated the distribution of each topic in the four time periods of negative mood (as shown in Figure 10). Low periods 1 and 2 were related to the politicization of the vaccine approval process: the number of tweets related to topic 4 in negative sentiment reached 22.77% on August 2; and the number of tweets related to topic 4 in negative sentiment reached 21.12% on August 22. In addition, the low period of 2 (August 22) was also related to topic 1. The negative sentiment in that period was mainly in two aspects: first, opponents' dissatisfaction with preventive and control measures such as wearing masks, herd immunization, and blockade; and second, supporters' dissatisfaction with some groups' violation of preventive measures. The emergence of trough periods 3 and 4 was associated with the suspension of vaccine clinical trials: the number of tweets related to topic 3 (*N* = 167) reached 51.38% in the negative sentiment on September 9; and the number of tweets related to topic 3 (*N* = 127) reached 53.14% in the negative sentiment on October 13.

Figure 11 reflects the daily trends of each type of sentiment, and we can find that the trends of negative, positive, and neutral sentiment behave in a similar way. The two obvious peaks are on August 11 and October 22, which correlate with the number of tweets on that day.

Figures 12 and 13 reflect tweets' distribution on each topic in positive and negative sentiment. It can be discovered that the two peaks in positive sentiment occurred on August 11 and October 22, respectively. The August 11 peak was associated with Russia's approval of the world's first COVID-19 vaccine; the October 22 peak was associated with the BJP's vaccine promise. The two peaks in negative sentiment that occurred on September 9 and October 13 were both associated with the suspension of vaccine trials.

## 4. Discussion

### 4.1. Principal Finding

The above study data can be used to explain the public response to the COVID-19 vaccine during the pandemic. Through textual analysis, we found that public discussion of the COVID-19 vaccine focused on 11 topics. Among them, the public paid the highest attention to the clinical trials of the vaccine, which reflected the public's psychological expectation of the vaccine. These 11 topics can be further divided into four themes: concerns about the COVID-19 epidemic; vaccine development, production, and distribution; the control of the epidemic before obtaining the vaccine; and knowledge or information related to the safety and efficacy of the vaccine.

From the temporal trends of the different topics, this study found four peaks in the discussion of vaccines. In addition to being associated with specific events (e.g., approval of the world's first vaccine in Russia; suspension of clinical trials for the AstraZeneca vaccine, etc.), these four peaks are also associated with the “Fresh start effect.” This suggests that public opinion is more likely to reach peak if the event of public interest occurs at the beginning of the week. In addition, we identified a number of potential factors that could threaten future vaccination rates, including vaccine nationalism, the politicization of the vaccine approval process, vaccine confidence crisis, vaccine hesitancy, vaccine rumors, and vaccine fundamentalism. These factors primarily affect vaccine distribution and public acceptance of vaccines. COVID-19 has developed into a global public health emergencyand increased the need for global efforts and cooperation. Vaccine nationalism has led to the inequitable distribution of vaccines around the world, with some poor countries, rural areas, and vulnerable populations unable to access vaccines timely. Related rumors do not only include vaccine-related rumors (e.g., that vaccines may alter a person's DNA), but also other immunization-related rumors (e.g., that coal miners and smokers are immune to COVID-19). The proliferation of these rumors on social media has reduced public recognition and acceptance of the vaccine, and caused the public to show hesitation or even outright refusal in terms of vaccination. The fear that the approval of the vaccine would be interfered with by political factors, in turn, reduced confidence in the vaccine. In contrast, endorsement from Dr. Fauci increases public trust in the vaccine, which is consistent with the findings of Bokemper et al. [31]. Although there is little discussion of Vaccine Fundamentalism in the tweets, it should also be of concern. The study from Drew shows that a high percentage of Christian fundamentalists in the United States show hesitation or even opposition to vaccines [32]; Łowicki et al. also confirm a positive correlation between religious fundamentalism and COVID-19 conspiracy beliefs [33]. In addition, we should also be alert to the pressures that a dual epidemic puts on the public health system before accessing the vaccine.

In terms of sentiment, overall there is more positive than negative and neutral. By analyzing the temporal trends, we identified four distinct periods of low sentiment. The emergence of these trough periods is mainly related to the suspension of vaccine trials, the politicization of the vaccine approval process, and COVID-19 prevention and control measures. Finally, we analyzed the temporal trends of positive and negative sentiments under different topics and found that the emergence of two peaks in positive sentiments was related to the Russian approval of the COVID-19 vaccine and the BJP's vaccine supply commitment, respectively; and the emergence of two peaks in negative sentiments was related to the suspension of vaccine experiments. In summary, the politicization of the vaccine approval process, suspension of vaccine experiments, and social measures to control the epidemic are highly likely to trigger negative public sentiment; whereas information related to successful vaccine development and supply increases positive public sentiment.

### 4.2. Practical Implications

For government departments and the public, social media is a convenient communication channel that can help policymakers better understand the public's response to the COVID-19 vaccine. These findings can help policymakers develop more accurate public health policies, reduce negative public sentiment during pandemics, properly guide the public to build up their knowledge and attitude toward the vaccine, and increase vaccination rates. Through analyzing, we found that public reaction to vaccines is a dynamic process, so the government's understanding of public perceptions and attitudes should also be a dynamic process. Government departments or policymakers should continuously adjust public health policies according to public reactions in order to improve the effectiveness of policy implementation. Tuesday is the peak of public discussion, so government and policymakers can start the week by announcing positive news and policy information related to vaccines in order to draw more attention to them. While the public expresses distrust of political leaders, it shows a high level of trust in scientists and expresses concern about the vaccine review process. Thus, policymakers need to make the vaccine review process public and use the role of scientists in communicating with the public to increase public trust in vaccines. International organizations (e.g., World Health Organization) or regional organizations (e.g., European Union) should play a role in the equitable distribution of vaccines to eliminate the threat of vaccine nationalism. Rumors on social platforms are also an important aspect that cannot be ignored, for which platforms and governments should work together to establish rumor verification mechanisms to combat false information and guide the public to build correct knowledge about vaccines. Since in most cases there is a close relationship between outbreaks of mass actions and negative sentiment, policymakers should dynamically assess changes in public sentiment and gain insight into specific events that lead to negative public sentiment in order to avoid outbreaks of vicious mass events. In addition, we also found that the public is also particularly concerned about the potential hazards of twindemic before vaccination, so it is important for policymakers to pay attention to and prepare for the prevention of other epidemic outbreaks (e.g., seasonal influenza) in advance during COVID-19 to reduce the stress of dual epidemics.

### 4.3. Limitations

There are several limitations to this study. First, we cannot obtain any information about deleted tweets as well as logouts due to the influence of Twitter policies. Second, we were unable to conduct an in-depth analysis of the geospatial characteristics of topics and sentiments due to the unavailability of geographic location information of tweets. Third, although this study identified the potential threat factors such as rumors, no targeted analysis of tweets about rumors was conducted, which led us to possibly not know the topic distribution and sentiment distribution of these rumors. Future studies can therefore be conducted with targeted analyses of relevant topics to help decision makers have a more comprehensive understanding of them.

## Figures and Tables

**Figure 1:** Timeline of tweets.

**Figure 2:** Trends in the number of tweets.

**Figure 3:** *N*-grams. (a) Top unigrams. (b) Top bigrams.

**Figure 4:** Word cloud map.

**Figure 5:** Consistency score.

**Figure 6:** Probability distribution of key terms under different topics.

**Figure 7:** The frequency distribution of tweets corresponding to each topic.

**Figure 8:** Time trends of the number of topics.

**Figure 9:** Time trends in sentiment.

**Figure 10:** Percentage distribution of topics under different peak periods.

**Figure 11:** Time trends of tweets in different sentiments.

**Figure 12:** The trend of the number of tweets corresponding to different topics in positive sentiment.

**Figure 13:** The trend of the number of tweets corresponding to different topics in negative sentiment.

**Table 1:** Date with the highest number of tweets.

	Date	Number of tweets
1	2020/8/11	1,411
2	2020/10/22	1,215
3	2020/9/9	931
4	2020/9/8	794
5	2020/9/16	774
6	2020/9/17	683
7	2020/10/13	677
8	2020/9/3	656
9	2020/8/12	638
10	2020/9/4	588

**Table 2:** The topics and themes in tweet.

Topic	Fifteen most common term	Theme
Topic 0	Health, pandemic, global, public, ensure, include, part, effort, access, support, fight, expert, response, lead, group	Theme 2
Topic 1	Virus, time, spread, infection, mask, patient, immunity, population, disease, control, show, kill, close, long, rate	Theme 3
Topic 2	Read, research, development, late, great, live, update, question, talk, join, share, discuss, watch, learn, challenge	Theme 4
Topic 3	Trial, clinical, phase, candidate, study, volunteer, start, early, AstraZeneca, human, begin, result, show, pause, participant	Theme 2
Topic 4	Make, trump, election, trust, science, rush, official, top, speed, push, big, explain, clear, pay, political	Theme 4
Topic 5	Plan, end, government, state, ready, free, announce, dose, potential, sign, promise, provide, deal, supply, distribution	Theme 2
Topic 6	Year, flu, find, people, important, protect, good, risk, covid, child, shot, time, prevent, vaccinate, increase	Theme 1
Topic 7	Test, give, people, back, life, hope, thing, care, call, school, lie, cure, vote, positive, open	Theme 3
Topic 8	Coronavirus, news, safety, race, datum, receive, treatment, Russian, approval, follow, drug, base, good, release, expect	Theme 4
Topic 9	Covid, people, case, day, report, month, death, week, die, wait, stop, high, happen, strategy, bad	Theme 1
Topic 10	Vaccine, develop, world, work, safe, country, effective, covid, scientist, approve, produce, create, make, deliver, development	Theme 2

^∗^Notice: Theme 1: concerns about COVID-19; Theme 2: concerns about vaccine development, production, and distribution; Theme 3: how to control COVID-19 before obtaining the vaccine; Theme 4: concerns about knowledge or information of vaccine safety and efficacy.

## Data Availability

Data presented in this study are available from the authors.
